The article "Systematic Evaluation of the Effect of Bedside Ward Round Checklist on Clinical Outcomes of Critical Patients" was published in 2021. Journal: J Healthc Eng.

# Systematic Evaluation of the Effect of Bedside Ward Round Checklist on Clinical Outcomes of Critical Patients

**DOI:** 10.1155/2021/8105516

**Published:** 2021-12-15

**Authors:** Xuemin Wen, YuXiang Wen, Ge Wang, Hui Li, Hong Zuo

**Affiliations:** ^1^Department of Nursing, First Affiliated Hospital of Chongqing Medical University, Chongqing, China; ^2^Chongqing Medical School, Chongqing, China; ^3^Department of Hematology, First Affiliated Hospital of Chongqing Medical University, Chongqing, China; ^4^Department of Nephrology, First Affiliated Hospital of Chongqing Medical University, Chongqing, China

## Abstract

**Objective:**

To systematically evaluate the effect of bedside ward round checklists on the clinical outcomes of critical patients and thus provide a scientific and rational basis for decision-making in its clinical application.

**Methods:**

PubMed, EMBASE, Web of Science, Cochrane Library, CNKI, and Wanfang databases were searched to collect the literature studies about randomized controlled trials (RCTs) and cohort studies involving the effect of bedside ward round checklists on the clinical outcomes of critical patients, and the retrieval time limit was from the establishment of the database to August 2019. After two researchers independently screened the literature studies, extracted the literature data, and evaluated the risk of bias in included studies, meta-analysis was carried out by using Stata 12.0 software.

**Results:**

Two RCTs and nine cohort studies were included in this study. The results of meta-analysis showed that compared with the ordinary bedside ward round, the application of checklist in bedside ward round could shorten the ICU hospitalization time (standardized mean difference (SMD) = – 0.37, 95% CI (– 0.78, 0.04), *P* ≤ 0.001) and mechanical ventilation time (SMD = – 0.24, 95% CI (– 0.44, −0.04), *P* = 0.037) and reduce the incidence of ventilator-associated pneumonia (VAP) (SMD = 0.61, 95% CI (0.38, 0.99), *P* = 0.057) in critical patients. However, there were no significant differences in central venous catheter (CVC) retention time and incidence and mortality of deep venous thrombosis (DVT) between ordinary ward round and bedside ward round checklist.

**Conclusion:**

The existing evidence shows that compared with the ordinary ward round, the application of bedside ward round checklists can shorten ICU hospitalization time and mechanical ventilation time and reduce VAP incidence and ICU mortality in critical patients. However, due to the limitations of the quality of the included studies, the above conclusions need to be verified with more high-quality studies.

## 1. Introduction

The condition in critical patients is complex, and multiple parallel treatment and nursing processes are being carried out. Insufficient process goal setting will directly affect the implementation of clinical decision-making. Bedside ward round is a communication mechanism for joint decision-making by both doctors and nurses [1]. Due to the area and time limitations, fast information access is particularly important in bedside ward round. In recent years, domestic and foreign scholars have found that checklists, as a process management optimization tool, have obvious utility values in ICU quality improvement, such as checklists for critical patient transfer [2, 3], surgical safety verification [3, 4], and ICU visitation management [5, 6]. A concise and clear “inventory checklist” can be used to reflect the changes in process key indicators and quickly project obstacle factors in quality control to managers [7]. However, the roles of the checklists in the studies on the application of bedside ward round for critical patients remain unclear. Although the checklist can improve the compliance of medical staff to clinical practice standards and reduce the incidence of adverse events in process management [8], previous studies at home and abroad showed that the bedside ward round checklists, which are not designed solely based on evidences, have no unified standard for the feasibility and effectiveness of their examination items. It is still controversial whether the application of bedside ward round checklists can ultimately improve the clinical outcome of critical patients, and currently, there is no comprehensive systematic evaluation. This study systematically evaluated the effect of bedside ward round checklists on the clinical outcome of critical patients, assessed the decision-making information needs of critical patients on bedside ward rounds, and further explored the timing and process management for the application of ICU bedside ward round checklists, so as to provide a decision-making basis for clinical evidence-based practice in the future.

The article "Systematic Evaluation of the Effect of Bedside Ward Round Checklist on Clinical Outcomes of Critical Patients" was published in 2021. Journal: J Healthc Eng.

## 2. Data and methods

### 2.1. Inclusion and Exclusion Criteria

#### 2.1.1. Inclusion Criteria

Inclusion criteria were as follows: ① study type: randomized controlled trial (RCT), cohort study; ② study subjects: ICU inpatients with complete case data and age ≥18 years; ③ intervening measures: the checklist was applied in bedside ward round in the test group, and ordinary bedside ward round was carried out in the control group; and ④ outcome indicators: there was at least one observation indicator in the study results, including ICU hospitalization time, CVC retention time, mechanical ventilation time, incidence of VAP, incidence of DVT, and mortality of ICU patients.

#### 2.1.2. Exclusion Criteria

Exclusion criteria were as follows: ① repeatedly published studies; ② studies with incomplete baseline data; ③ studies with incomplete summary information; and ④ conference papers, reviews, and case reports

### 2.2. Literature Retrieval Strategy

PubMed, EMBASE, Web of Science, Cochrane Library, CNKI, and Wanfang databases were searched to collect the literature studies about randomized controlled trials (RCTs) and cohort studies involving the effect of bedside ward rounds on the clinical outcomes of critical patients, and the retrieval time limit was from the establishment of the database to August 2019. The retrieval was carried out by combining subject words with free words. English search terms included intensive care unit, bedside ward rounds, ICU rounds, ICU bedside ward rounds, checklist, and ICU daily bedside ward round checklist; and Chinese search terms included the bedside ward round, ICU ward round, ICU bedside ward round, list, and ICU daily ward round list.

### 2.3. Literature Quality Evaluation

The quality evaluation of each RCT shall be independently evaluated by two evaluators according to the quality evaluation standards in the Cochrane system evaluator manual. In case of differences, the third evaluator shall intervene and reach a consensus to form a final decision [9]. Criteria include the following: ① generation of random sequence (selection bias); ② blind allocation (selection bias); ③ all study participants and personnel were blinded (implementation bias); ④ the results were evaluated by blind method (observation bias); ⑤ results data integrity (loss of follow-up bias); ⑥ select reports (report bias); and ⑦ others.

### 2.4. Literature Screening, Data Extraction, and Bias Risk Assessment of Included Studies

Two researchers independently screened the literature studies, extracted the data, and performed a crosscheck. A third independent researcher was consulted to achieve final consensus in case of disagreement, and the authors were contacted to supplement the missing data as far as possible. During literature screening, titles and abstracts should be read at first. After obviously irrelevant literature studies were excluded, full texts should be further read to determine whether remaining literature studies were finally included. A self-made data extraction table was used to extract relevant information from the literature studies that met the inclusion criteria. The data to be extracted mainly included the following: ① basic information of included studies, such as study topic, first author, publication time, and study type; ② baseline characteristics of study subjects, such as sample size, age, and gender; ③ specific details of intervening measures; ④ key elements of bias risk assessment; and ⑤ outcome indicators and outcome measurement data, which were concerned. The bias risk of included RCTs was evaluated by using an evaluation tool from JBI Evidence-Based Health Care Center in Australia. The bias risk of included cohort studies was evaluated by using the Newcastle–Ottawa scale (NOS).

The article "Systematic Evaluation of the Effect of Bedside Ward Round Checklist on Clinical Outcomes of Critical Patients" was published in 2021. Journal: J Healthc Eng.

### 2.5. Bias Risk Assessment

Two evaluators used the bias risk assessment tool for RCT provided by the Cochrane manual to evaluate the bias risk of the included studies.

### 2.6. Statistical Analysis

Statistical 12.0 software was used for meta-analysis. The mean difference (MD) was used as the effect indicator for continuous data, and the odds ratio (OR) was used as the effect size for categorical data. Point estimate and 95% CI were given for each effect size. Statistical heterogeneity among the study results was assessed by a *χ*^2^ test (test level *α* = 0.1), and the heterogeneity was assessed by the combined use of *χ*^2^ and I^2^ tests. If there was no statistical heterogeneity among the studies, the fixed effect model was used for meta-analysis; if there was a statistical heterogeneity among studies, the sources of heterogeneity were further analyzed. After the effect of obvious clinical heterogeneity was excluded, a random effect model was used for meta-analysis. If there was a significant clinical heterogeneity among the study results, subgroup analysis or sensitivity analysis should be performed. The inspection level of meta-analysis was set as *α* = 0.05.

## 3. Results

### 3.1. Literature Screening Process and Results

A total of 11 literature studies were included in this study, including 8 in English and 3 in Chinese. The literature screening process and results are shown in Figure 1, basic features of included studies are shown in Table 1, and the literature quality evaluation is shown in Table 2.

### 3.2. Basic Features of the Included Studies

See Table 1

### 3.3. Assessment of Risk of Bias in Included Studies

The assessment of risk of bias in included RCTs is shown in Table 2; the assessment of risk of bias in included cohort studies is in Table 3.

① Was the random grouping method really adopted for the study subjects? ② Was the allocation concealment done? ③ Was the baseline data comparable between groups? ④ Were the study subjects blinded? ⑤ Were the interveners blinded? ⑥ Were the result evaluators blinded? ⑦ Except for the intervening measures to be verified, were other measures accepted equally by each group?⑧ Was the follow-up completed? If not, were some measures taken to deal with the loss of follow-up? ⑨ Were all randomly assigned subjects included in the outcome analysis? ⑩ Were the outcome indicators of subjects in each group evaluated in the same way? ⑪ Was the evaluation method of outcome indicators credible? ⑫ Was the data analysis method appropriate? And ⑬ Was the study design reasonable?

①There was population representativeness in the cohort group; ② the samples in the control group were from the same population as those in the cohort group; ③ the methods were used for determining exposure factors; ④ there were no outcome indicators to be observed at the beginning of the study; ⑤ the most important confounding factors were controlled in the study; ⑥ other confounding factors were controlled in the study; ⑦ evaluation of outcomes: whether the scoring of the results was sufficient in the study; ⑧ whether the follow-up time was long enough; and ⑨ whether the follow-up in the cohort group and the control group was sufficient.

The article "Systematic Evaluation of the Effect of Bedside Ward Round Checklist on Clinical Outcomes of Critical Patients" was published in 2021. Journal: J Healthc Eng.

### 3.4. Meta-Analysis Results

#### 3.4.1. ICU Hospitalization Time of Patients

This outcome indicator was reported in 10 studies [1, 3, 5, 8, 10–12]. The results of meta-analysis of the random effect model showed that the application of checklist in bedside ward round could reduce the ICU hospitalization time compared with ordinary bedside ward round [standardized mean difference (SMD) = –0.37, 95%CI (–0.78, 0.04), *P* ≤ 0.001], and the difference was statistically significant. Further subgroup analysis was conducted according to different study designs. The results showed that compared with the ordinary ward round, the application of the checklist in bedside ward round in the RCT subgroup could significantly reduce the ICU hospitalization time of patients [SMD = –0.82, 95%CI (–1.47, –0.16),*P* ≤ 0.001], while the decrease in ICU hospitalization time in the cohort study subgroup was not significant [SMD = –0.22, 95%CI (–0.40, –0.05), *P* ≤ 0.001], but the difference was still statistically significant (Figure 2).

#### 3.4.2. CVC Retention Time

The result showed that only 2 cohort studies were included [3, 12]. The results of fixed effect model meta-analysis showed that there was no significant difference in CVC retention time between application of the checklist in ward rounds and ordinary ward rounds (MD = –0.52, 95% CI (–0.72,–0.31), *P* = 0.334) (Figure 3).

#### 3.4.3. Mechanical Ventilation Time

This outcome indicator was reported in 4 studies [7, 10–12]. The results of the meta-analysis of the random effect model showed that compared with ordinary ward rounds, the application of the checklist in ward rounds could reduce the mechanical ventilation time (SMD = −0.24, 95% CI (−0.44, −0.04), *P* = 0.037), and the difference was statistically significant (Figure 4).

The article "Systematic Evaluation of the Effect of Bedside Ward Round Checklist on Clinical Outcomes of Critical Patients" was published in 2021. Journal: J Healthc Eng.

#### 3.4.4. VAP Incidence

This outcome indicator was reported in 5 studies [1, 2, 8, 10, 11]. The results of meta-analysis of the random effect model showed that the application of the checklist in ward rounds could reduce the VAP incidence compared with ordinary ward rounds (SMD = 0.61, 95% CI (0.38,0.99), *P* = 0.057), but the difference was not statistically significant (Figure 5).

#### 3.4.5. DVT Incidence

This outcome indicator was only reported in two included cohort studies [3, 6]. The results of the fixed effect model meta-analysis showed that there was no significant difference in the DVT incidence between the application of the checklist in ward rounds and ordinary ward rounds (MD = −0.52, 95% CI (−0.72, −0.31), *P* < 0.334) (Figure 6).

#### 3.4.6. Patient Mortality

The outcome indicator was reported in 6 included studies [2, 3, 6, 8, 11, 12], of which 4 were cohort studies and 2 were RCTs. The results of the heterogeneity test showed that *P* = <0.1, so the random effect model was adopted. The meta-analysis results showed that although the application of checklist in ward rounds could reduce the mortality of patients compared with ordinary ward rounds (OR = 0.72, 95% CI (0.50, 1.03)), the difference was not statistically significant (*P* > 0.05). Further subgroup analysis was conducted according to different study designs. The results showed that although the application of the checklist in ward rounds in RCTs could increase the mortality of patients compared with ordinary ward rounds (OR = 1.04, 95% CI (0.94, 1.16)), the difference was not statistically significant (*P* > 0.05). The application of the checklist in ward rounds in cohort studies could reduce the mortality of patients compared with ordinary ward rounds (OR = 0.60, 95% CI (0.39, 0.91)), and the difference was statistically significant (*P* < 0.05) (Figure 7).

## 4. Discussion

### 4.1. Bedside Ward Round Checklist Is Conducive to Improving the Clinical Outcome of Critical Patients

In the bedside ward rounds of critical patients, the checklist can be used to quickly identify the the focus of quality inspection [8]. Nine cohort studies [8, 10, 14, 16, 18] and two RCTs [15, 17] were included in this study, and the results showed that the application of the bedside ward round checklist could reduce the incidence of unexpected adverse events in critical patients and play a positive role in improving the prognosis of critical patients, of which 2 cohort studies [11, 13] revealed that the application of the bedside ward round checklist can reduce the incidence of DVT in critical patients, 1 RCT [16] and 5 cohort studies [8, 9, 11, 16, 17] showed that the bedside ward round checklist is conducive to reducing ICU hospitalization time, and 5 clinical studies [1, 2, 8, 10, 11]showed that ICU critically ill patients need to be treated with mechanical ventilation. Due to long-term hospitalization in ICU, the risk of infection will increase. The bedside ward round checklist provides patients with satisfactory and real-time clinical services from a comprehensive perspective. It can reduce the incidence of VAP complications in ICU critically ill patients and apply it to clinical nursing of ICU critically ill patients. It plays an important role in promoting the rehabilitation of patients. Because the proportion of ICU patients using mechanical ventilation is high, and ICU patients are in critical condition, if routine nursing is given, it is easy to increase the incidence of VAP, which increases the mortality of patients and prolongs the length of hospital stay. Two cohort studies [3, 12] showed that the special nursing of bedside ward round checklist strategy can effectively reduce the incidence of central venous catheter-related bloodstream infection, shorten the length of hospital stay, make the patient's rehabilitation process smooth, and reduce the medical burden and economic burden. A multicenter cohort study in Australia [14] found that the implementation of the bedside ward round checklist can effectively reduce the difference between evidence-based treatment and practice, and the checklist demonstrates dynamic changes in disease, whereby individualized treatment plans can be formulated, which effectively reduces the mechanical ventilation time for ICU patients and highlights the advantageous effect of the ward round checklist on the clinical outcome of critical patients. However, the long-term effects of the ward round checklist on the quality of life of critical patients still need to be further verified and discussed. The application of the bedside ward round checklist will help to carry out targeted clinical nursing measures, promote blood circulation, reduce ischemia and hypoxia caused by long-term lying in bed and long-term compression of local tissues, and reduce the incidence of ventilator-associated pneumonia due to too long mechanical ventilation time. The infection caused by the indwelling time of central venous catheter, the incidence of deep venous thrombosis, and complications. This method can reduce nursing risk, ensure patient safety, and promote the continuous improvement of nursing quality, so as to make diagnosis and treatment as soon as possible, so as to improve the prognosis of patients.

The article "Systematic Evaluation of the Effect of Bedside Ward Round Checklist on Clinical Outcomes of Critical Patients" was published in 2021. Journal: J Healthc Eng.

### 4.2. Sufficient Evidences Are Still Needed to Fully Promote the Bedside Ward Round Checklist in ICU

International attention is increasingly paid to the quality and safety of intensive care practice. In order to optimize the strategy of the bedside ward round quality management mode for critical patients, we must consider the effects of comprehensive factors on the implementation of the bedside ward round checklist. Although bedside ward round checklists were used in all literature studies included in this study, their using effects were still different due to the limitations of multiple factors, such as patient population characteristics, hospital environment, medical staff, and process optimization measures. Most studies lacked a detailed description of the characteristics of the included and excluded population and ignored the heterogeneity of population characteristics. Only in one study, it was mentioned that the included population was trauma ICU patients, and the injury severity score (ISS) was compared between two groups of patients [8]; in a domestic RCT [18], the authors used CERTAIN electronic checklist developed by Mayo Clinic in the United States after being converted into Chinese; the results showed that the ICU hospitalization time, mechanical ventilation time, and VAP incidence were reduced, but there was no significant difference in 28d mortality, which may be related to the small sample size, cultural environment differences between at home and abroad, and the influencing factors of primary disease; although the structured bedside ward round checklist can prevent the occurrence of adverse events during treatment and nursing, after the authors carefully verified the items in the checklist in a cohort study [14], the author accidentally found that only 3 of the 9 nursing process indicators were applicable to the morning bedside ward rounds; it was found in the results of 1 RCT [15] that the introduction of process indicators recommended in the guidelines as review items in the checklist had no significant effect on the mortality of ICU patients, which reminds us that we should further clarify the correlation between the checklist item setting and the currently commonly used clinical process indicators. The population selection bias, sample size limitation, and the lack of representativeness of process indicators restrict the popularization of the checklist, so it is necessary to individually screen and appropriately improve the contents of the checklist. When extrapolating the short-term results of the study report into the predicted long-term effectiveness, we must pay attention to the scientificity and accuracy of the result observation. The setting of observation period length of clinical outcomes was different in all included literature studies in this study, the maximum time interval from baseline to intervention was 13 months [10], and the time setting basis is not clearly explained in the article. Although process optimization is carried out, some prognostic indicators are improved, but not all problems of critical patients are solved in bedside ward rounds. The differences in intervention timing and observation window settings still make it impossible for us to determine whether the bedside ward round checklist can become an independent factor affecting the clinical outcome of critical patients. Changes in the study design and limitations in the reports affect the summary of interaction trends between intervention measures and outcomes. Therefore, more high-quality and large-sample evidences are still needed to confirm the effectiveness of reasonably constructed bedside ward round checklist and facilitate its comprehensive popularization in clinical practice.

The article "Systematic Evaluation of the Effect of Bedside Ward Round Checklist on Clinical Outcomes of Critical Patients" was published in 2021. Journal: J Healthc Eng.

### 4.3. Limitations of This Study

The number of patients included in each study was small; the contents of bedside ward round checklists in included studies were not exactly the same; due to the limitation of the number of literature studies, only two RCT studies are included. In the future, it will be needed to carry out multicenter and strict clinical RCTs, scientifically set the contents of bedside ward round checklist, strictly control the start time, and formulate relatively unified bedside ward round checklist for critical patients in terms of quality control and effectiveness of observation time interval.

## 5. Conclusion

Bedside ward round checklist plays a positive role in the clinical outcome of critical patients, but further discussion and verification are still needed for comprehensive promotion of the bedside ward round checklist. The correlation between the checklist response and the actual clinical treatment should be considered to improve the consistency between the treatment plan adjustment and the bedside ward round checklist response.

## Figures and Tables

**Figure 1:** Literature screening process.

**Figure 2:** Meta-analysis of the effect of ward round checklist on ICU hospitalization time compared with ordinary ward round.

**Figure 3:** Meta-analysis of the effect of application of the checklist in ward rounds on CVC retention time in patients compared with ordinary ward rounds.

**Figure 4:** Meta-analysis of the effect of application of the checklist in ward rounds on mechanical ventilation time in patients compared with ordinary ward rounds.

**Figure 5:** Meta-analysis of the effect of application of the checklist in ward rounds on the incidence of VAP compared with ordinary ward rounds.

The article "Systematic Evaluation of the Effect of Bedside Ward Round Checklist on Clinical Outcomes of Critical Patients" was published in 2021. Journal: J Healthc Eng.

**Figure 6:** Meta-analysis of the effect of application of the checklist in ward rounds on the incidence of DVT compared with ordinary ward rounds.

**Figure 7:** Meta-analysis of the effect of the application of the checklist in ward rounds on the mortality of patients compared with ordinary ward rounds.

**Table 1:** Basic features of the included studies.

Included studies	Study type	Cases (T/C)	Age（T/C）, years	Intervening measure			Outcome indicator
				T	C				
DuBose et al. [10]	Cohort study	570/577	39.0 ± 21.1/39.4 ± 20.6	Bedside ward round checklist		Ordinary ward round		①④⑥
Stone et al. [8]	Cohort study	89/85	47.3 ± 23.7/44.4 ± 19.7	Bedside ward round checklist		Ordinary ward round		①③④
Weiss et al. [11]	Cohort study	140/125	58.5 ± 17.8/57.3 ± 17.8	Bedside ward round checklist		Ordinary ward round		①②③⑤⑥
Ilanet al. [12]	Cohort study	110/81	65 ± 16/63 ± 17	Bedside ward round checklist		Ordinary ward round		②
Haitham 2014	Cohort study	130/216	57.33 ± 18.32/54.88 ± 18.28	Bedside ward round checklist		Ordinary ward round		①③
Reiff et al. [13]	Cohort study	1185/1136	45.1 ± 19.3/43.5 ± 18.8	Bedside ward round checklist		Ordinary ward round		①③⑤⑥
Conroy et al. [14]	Cohort study	152/141	57 ± 18/57 ± 21	Bedside ward round checklist		Ordinary ward round		①③
Cavalcanti et al. [15]	RCT	3327/3434	59.1 ± 19.2/60.0 ± 18.8	Bedside ward round checklist		Ordinary ward round		①③④⑥
Chen et al. [16]	Cohort study	1172/886	63.65 ± 17.67/64.01 ± 16.12	Bedside ward round checklist		Ordinary ward round		①③④
Wen et al. [17]	Cohort study	50/50	58.46 ± 15.69/60.66 ± 13.18	Bedside ward round checklist		Ordinary ward round		①②③⑥
Fan et al. [18]	RCT	87/86	54.75 ± 20.77/50.80 ± 18.64	Bedside ward round checklist		Ordinary ward round		①③④⑥

T: test group; C: control group; ① ICU hospitalization time; ② central venous catheter (CVC) retention time; ③ mechanical ventilation time; ④ incidence of ventilator-associated pneumonia (VAP); ⑤ incidence of deep venous thrombosis (DVT); and ⑥ ICU patient mortality.

**Table 2:** Assessment of risk of bias in included RCTs.

Included studies	①	②	③	④	⑤	⑥	⑦	⑧	⑨	⑩	⑪	⑫	⑬
Cavalcanti et al [15]	Yes	Yes	Yes	Yes	Yes	Yes	Yes	Yes	Yes	Yes	Yes	Yes	Yes
Fan et al. [18]	Yes	Yes	Yes	Yes	Unclear	Unclear	Yes	Yes	Yes	Yes	Yes	Yes	Yes

**Table 3:** Assessment of risk of bias in included cohort studies.

Cohort study	①	②	③	④	⑤	⑥	⑦	⑧	⑨	Total NOS score
DuBose et al. [10]	1	1	1	0	1	1	1	1	1	8
Stone et al. [8]	1	1	1	1	1	1	1	1	1	9
Weiss et al. [11]	1	1	1	1	1	1	1	1	1	9
Ilanet al. [12]	1	1	1	0	1	1	1	1	1	8
Haitham 2014	1	1	1	1	1	1	0	1	1	8
Reiff et al. [13]	1	1	1	1	1	1	1	1	0	8
Conroy et al. [14]	1	1	1	1	1	1	1	1	0	8
Cavalcanti et al. [15]	1	1	1	1	1	1	0	0	0	6
Chen et al. [16]	1	1	1	1	1	1	0	0	0	6

The article "Systematic Evaluation of the Effect of Bedside Ward Round Checklist on Clinical Outcomes of Critical Patients" was published in 2021. Journal: J Healthc Eng.

## Data Availability

The simulation experiment data used to support the findings of this study are available from the corresponding author upon request.
